The article "Influence of Oxytocin Usage and Dose Difference During Delivery on Pregnancy Outcome of VBAC Pregnant Women" was retracted in 2023. Reasons: unreliable results or conclusions; lack of ethics approval or compliance; concerns about the data; concerns about the peer review.

# Influence of Oxytocin Usage and Dose Difference During Delivery on Pregnancy Outcome of VBAC Pregnant Women

**DOI:** 10.1155/2022/6038924

**Published:** 2022-08-09

**Authors:** Zhuo Yuan, Lei Hu, Wanying Li, Shuo Zhou, Nana Zhu, Qi Lv

**Affiliations:** Three Treatment Areas of Obstetrics, Changchun Maternity Hospital, Changchun 130042, China

## Abstract

In order to explore the influence of oxytocin usage and dose difference during delivery on the pregnancy outcome of VBAC pregnant women, the clinical data of 166 VBAC pregnant women from January 2017 to March 2020 are retrospectively analyzed. All women are divided into different groups according to the usage of oxytocin during delivery and the oxytocin dose difference. Binary logistic regression is used to analyze the factors affecting the pregnancy outcome of pregnant women with VBAC. The gestational weeks and the thickness of the lower uterine segment in the oxytocin group are significantly more than those in the nonoxytocin group (*P* < 0.05). The time of the first stage of labor, second stage of labor, and total stage of labor in the oxytocin group are significantly longer than the nonoxytocin group (*P* < 0.05). The proportion of entering NICU in the oxytocin group is significantly lower than the nonoxytocin group (*P* < 0.05). There is no significant difference in labor duration and pregnancy outcome between low-dose and medium-dose oxytocin groups. Binary logistic regression analysis shows that prenatal BMI <30 kg/cm^2^, gestational age ≤40 weeks, history of vaginal delivery, uterine expansion, and admission to hospital are the influencing factors for pregnancy success of pregnant women with VBAC. The usage of oxytocin in VBAC pregnant women during delivery may increase the duration of labor. For those with poor uterine contraction, oxytocin can be increased to 4∼18 mU/min to speed up the labor process, without increasing the risk of adverse pregnancy outcomes.

## 1. Introduction

In recent years, with the change of the fertility guidance policy and the implementation of the second child policy, the proportion of the second child-bearing age women has increased obviously [1]. Previous reports suggested that the cesarean section rate in different regions of China is between 40% and 55%. In recent years, more and more clinicians have begun to implement vaginal delivery for pregnant women with vaginal trial conditions after cesarean section, and accumulated rich clinical experience [2].

However, whether oxytocin can be given at a specific dose in VBAC pregnant women during delivery is not clear. In this study, we reviewed 166 cases of VBAC pregnant women from January 2017 to March 2020. The purpose of this study was to explore the effect of oxytocin use and dose difference on the pregnant outcome of VBAC pregnant women during delivery, according to whether oxytocin was used or not and different doses divided into groups.

The article "Influence of Oxytocin Usage and Dose Difference During Delivery on Pregnancy Outcome of VBAC Pregnant Women" was retracted in 2023. Reasons: unreliable results or conclusions; lack of ethics approval or compliance; concerns about the data; concerns about the peer review.

The rest of this paper is organized as follows: Section 2 discusses related work, followed by the data and method for oxytocin usage of VBAC pregnant women designed in Section 3. The results of this analysis are shown in Section 4.  Section 5 shows the discussion of results, and Section 6 concludes the paper with a summary and future research directions.

## 2. Related Work

There is no consensus on whether oxytocin can increase the risk of uterine rupture in pregnant women undergoing vaginal trial delivery after cesarean section [3]. Studies have shown that the use of oxytocin is closely related to the occurrence of uterine rupture during vaginal trial production after cesarean section. However, there was also a contrary view that there was no correlation between the two [4]. ACOG guidelines suggested that vaginal trial production should not be used as a contraindication for oxytocin. SOGC and RCOG also support this view [5].

Previous studies have found that some VBAC mothers have prolonged the labor process due to insufficient uterine contraction intensity, and oxytocin can effectively enhance uterine contraction and productivity, and accelerate the process of vaginal delivery [6]. Montoya-Williams et al. believed that some VBAC parturients have a prolonged labor process due to insufficient uterine contraction intensity, while the use of oxytocin can effectively enhance uterine contraction and productivity, and speed up the process of vaginal delivery. Some scholars have confirmed that the use of high-dose oxytocin is related to the risk of uterine rupture [7]. Although it is obvious that pregnant women can inject oxytocin intravenously during VBAC delivery, ACOG does not show the dose limit of oxytocin during uterine rupture and vaginal trial delivery [8]. Early studies showed that the peak dose of oxytocin in the medium-dose group was 18 *μ*M/min and no uterine rupture was found [9]. It is not recommended that pregnant women who become pregnant again after cesarean section should inject oxytocin intravenously for vaginal trial delivery. When the dilation of uterine orifice stops, artificial rupture of membrane should be preferred [10]. Hidalgo-Lopezosa et al. deem that the previous pregnancy history leads to the influence of uterine myometrium on hormone sensitivity, which makes the hormone sensitivity decrease in the second pregnancy. The effect can be achieved by increasing the dosage. It is not recommended that oxytocin should be given intravenously to pregnant women who are pregnant again after cesarean section for vaginal trial delivery. Artificial rupture of membrane should be the first choice when the dilatation of uterine orifice stops [10]. If oxytocin is needed during delivery, it is necessary to closely monitor the uterine contraction and fetal heart rate changes. If there is a risk of dystocia, it is recommended to give a low-dose oxytocin drip, and dynamically adjust the drip speed until effective uterine contraction occurs. After oxytocin administration, the frequency of uterine contraction should be no more than 4 times/10 min, and the maximum dosage of oxytocin should be no more than 20 mU/min. In addition, the dynamic evaluation of cervix should be strengthened during delivery, and the indications of cesarean section should be further expanded for those with poor progress of labor. Dynamic evaluation of cervix should be strengthened during delivery, and cesarean section indications should be further expanded for those with poor labor process [11].

The article "Influence of Oxytocin Usage and Dose Difference During Delivery on Pregnancy Outcome of VBAC Pregnant Women" was retracted in 2023. Reasons: unreliable results or conclusions; lack of ethics approval or compliance; concerns about the data; concerns about the peer review.

In the past, a large number of scholars at home and abroad conducted studies on the success factors of VBAC, and a large number of sample experiments showed that the success rate of VBAC trial delivery in pregnant women over 40 years old was significantly lower than that in pregnant women under 40 years old [12]. Studies have shown that the success rate of VBAC for pregnant women with uterine orifice opening >4 cm is significantly increased, and the larger the uterine orifice opening, the higher the success rate [13]. Gestational age ≤40 weeks is a factor influencing the success of VBAC. The longer gestational age is, the more likely it is to develop into macrofetus, so the success rate of VBAC is low [14, 15]. However, when cesarean section is performed again with a previous history of vaginal delivery, the pregnant women have good psychological preparation, have stronger confidence, and greater psychological support, and are more aware of the benefits of natural delivery, which is better for both themselves and the fetus than cesarean section, so the success rate of VBAC is significantly improved [16–19]. In terms of prenatal admission, the physiological hormone levels of pregnant women meet the requirements of natural clinical practice, so the success rate of VBAC can be improved.

## 3. Data and Method

### 3.1. Research Object

This study retrospectively analyzes the clinical data of 166 pregnant women with VBAC in our hospital from January 2017 to March 2020. Then, patients are divided into two groups according to whether oxytocin is used or not and the dose difference during delivery. The oxytocin dose subgroup includes the low-dose group and medium-dose group, which are given <4 mU/min and 4∼18 mU/min oxytocin, respectively.

The article "Influence of Oxytocin Usage and Dose Difference During Delivery on Pregnancy Outcome of VBAC Pregnant Women" was retracted in 2023. Reasons: unreliable results or conclusions; lack of ethics approval or compliance; concerns about the data; concerns about the peer review.

### 3.2. Inclusive Criteria and Exclusion Criteria

Inclusive criteria mainly include the following: (1) nonclassical cesarean section or T-shaped incision is used in the previous cesarean section. (2) Only one cesarean section is performed. (3) Transverse incision of the lower uterine segment. (4) The time from the last delivery is more than 18 months. (5) The clinical data are completed.

Exclusion criteria mainly include the following: (1) contraindications of vaginal delivery; (2) serious complications occur after the last cesarean section; (3) history of uterine rupture; (4) history of scar uterus surgery.

The design of the study protocol met the requirements of the Declaration of Helsinki, and the patients and their families have informed consent.

### 3.3. Methods

The vaginal trial delivery after cesarean section is evaluated by the obstetrician with the title of deputy senior or above, and the pregnant women and their families are still willing to accept the risk. If the indications of induced labor appear, they will be admitted to the hospital, and the mode of induced labor will be selected according to the Bishop score of the cervix. Among them, oxytocin intravenous drip for induction of labor is performed with patients whose B score is ≥6, while those with a B score < 6 receive water sac for ripening. All pregnant women should observe in the delivery room, open the venous channel after induction of labor and labor, and continuously monitor the fetal heart rate. In case of stagnation of labor, fetal distress, abnormal fetal heart rate, threatened uterine rupture, or family members, they should be transferred to cesarean section immediately [20]. For those with poor progress of labor, artificial rupture of membranes and intravenous drip of oxytocin are used to enhance the intensity of uterine contraction. Oxytocin is given by intravenous pump, i.e., 0.5% oxytocin 1 mU/min was given by pump, and the infusion rate should be ≤20 mU/min. For those who require labor analgesia, intraspinal analgesia is feasible. The indication of forceps delivery is that the opening of the uterine orifice is less than *S* + 2. It can be seen that in fetal distress, the time of the second stage of labor was more than 2 hours or the pregnant women need vaginal delivery.

### 3.4. Observation Index

The age, pregnancy time, delivery time, height, weight, gestational week, delivery mode, time from the last delivery, the use of oxytocin in the process of delivery, delivery time, and pregnancy outcome are recorded. The outcomes of pregnancy include midwifery, perineum injury, postpartum hemorrhage, fetal distress, neonatal asphyxia, and NICU entry. The specific standards refer to relevant literature [4]. A subgroup is established for the pregnancy outcomes of all pregnant women with VBAC included in this study. The differences in clinical data between the two groups are analyzed by univariate analysis, and the factors related to pregnancy success of pregnant women with VBAC are analyzed by binary logistic regression.

The article "Influence of Oxytocin Usage and Dose Difference During Delivery on Pregnancy Outcome of VBAC Pregnant Women" was retracted in 2023. Reasons: unreliable results or conclusions; lack of ethics approval or compliance; concerns about the data; concerns about the peer review.

### 3.5. Statistical Treatment

SPSS22.0 software is selected to process the data. The measurement data are compared by paired *t*-test and variance analysis, and data are expressed as $\bar{\chi }\pm S$. Comparison of counting data is evaluated by *χ*^2^ test or Fisher exact probability method, expressed as percentage (%). The factors related to the successful pregnancy of pregnant women with VBAC are analyzed by binary logistic regression. *P* < 0.05 is statistical significance in judging the difference.

## 4. Experimental Results

### 4.1. Comparison of Baseline Clinical Data between Oxytocin Group and Nonoxytocin Group

Table 1 shows the gestational age and the thickness of the lower uterine segment in the oxytocin group are significantly higher than those in the nonoxytocin group (*P* < 0.05). There is no significant difference in other baseline clinical data between the two groups (*P* > 0.05).

### 4.2. Comparison of Labor Process Time and Pregnancy Outcome between Oxytocin Group and Nonoxytocin Group

Second and total labor course of pregnant women in the group of oxytocin are significantly longer than those in the group without oxytocin (*P* < 0.05). The proportion of the patients who used oxytocin in NICU is significantly lower than that of the control group (*P* < 0.05), as shown in Table 2 and Figure 1.

### 4.3. Comparison of Labor Duration and Pregnancy Outcome in Different Oxytocin Dose Groups

There is no significant difference in labor duration and pregnancy outcome between low-dose and medium-dose oxytocin groups (*P* > 0.05), as shown in Table 3.

### 4.4. Univariate Analysis of Clinical Data Differences of VBAC Pregnant Women with Different Pregnancy Outcomes

There are no significant differences in age, incision scar length and birth weight between the two groups (*P* > 0.05). There are statistically significant differences in prenatal BMI, gestational age, history of vaginal delivery, degree of uterine orifice dilation, and admission to hospital (all *P* < 0.05), as shown in Table 4.

### 4.5. Binary Logistic Regression Analysis of Pregnant Women with VBAC Pregnancy Success Related Factors

The factors with *P* < 0.05 in result 4.4 are included as independent variables, and the pregnancy outcome of pregnant women with VBAC is included as dependent variables. Binary logistic regression analysis shows that prenatal BMI <30 kg/cm^2^, gestational age ≤40 weeks, history of vaginal delivery, uterine expansion, and admission to hospital are the influencing factors for pregnancy success of pregnant women with VBAC, as shown in Table 5 and Figure 2.

The article "Influence of Oxytocin Usage and Dose Difference During Delivery on Pregnancy Outcome of VBAC Pregnant Women" was retracted in 2023. Reasons: unreliable results or conclusions; lack of ethics approval or compliance; concerns about the data; concerns about the peer review.

## 5. Data Analysis and Result Discussion

There is no clear conclusion on whether oxytocin will increase the risk of uterine rupture in pregnant women who undergo vaginal trial after cesarean section. Previous studies have shown that there is a close correlation between the use of oxytocin and the occurrence of uterine rupture in the process of vaginal trial delivery after cesarean section. However, there is also a relative view that there is no correlation between the two. In this study, there is no uterine rupture in the group with or without oxytocin, so it is impossible to evaluate the effect of oxytocin on uterine rupture of pregnant women with vaginal trial delivery after cesarean section. Therefore, larger sample size and multicenter research are still needed.

There is no significant difference in the proportion of forceps delivery, perineal incision, postpartum hemorrhage, fetal distress, and neonatal asphyxia between the two groups. However, the duration of the first, second, and total stages of labor in the oxytocin group is significantly longer than that in the nonoxytocin group, suggesting that the use of oxytocin in the delivery process of VBAC pregnant women would not affect the maternal and infant outcomes, but may prolong the duration of labor. At the same time, there is no significant difference in labor time and pregnancy outcome between low-dose and medium-dose oxytocin groups, which confirmed that increasing the dropping speed and dose of oxytocin when necessary do not affect labor time and pregnancy outcome.

In addition, this study analyzed the influencing mechanism of pregnancy outcome of the included subjects. However, the results of this study are not reflected, which may be related to the small sample size of this study and the corresponding sample age. The results of this study showed that from univariate analysis of the success rate of VBAC, there were statistically significant differences between the VBAC group and the control group in prenatal BMI, gestational age, history of vaginal delivery, uterine dilation at admission, and admission to hospital during labor (*P* < 0.05). Multivariate analysis: prenatal BMI<30 kg/m^2^, gestational age ≤40 weeks, history of vaginal delivery, admission of uterine orifice dilation ≥6 cm, <6 years since the last cesarean section, and admission to labor all had an impact on the success rate of VBAC. Gestational age ≤40 weeks is a factor influencing the success of VBAC.

The article "Influence of Oxytocin Usage and Dose Difference During Delivery on Pregnancy Outcome of VBAC Pregnant Women" was retracted in 2023. Reasons: unreliable results or conclusions; lack of ethics approval or compliance; concerns about the data; concerns about the peer review.

## 6. Conclusion

In conclusion, the use of oxytocin in VBAC pregnant women may increase the duration of labor. For patients with poor uterine contraction, the dose of oxytocin can be increased to 4∼18 mU/min to accelerate the labor process, and it does not increase the risk of adverse pregnancy outcomes. A clinical study on the duration of labor of VBAC pregnant women shows that the duration of the active stage of labor, and the second stage of labor of this group was significantly longer than that of primipara but shorter than that of normal multipara, and the proportion of midwifery is also higher. However, this study did not pay attention to the relationship between the use of oxytocin and the duration of labor in VBAC pregnant women. Some scholars are worried about the risk of uterine rupture and suggest active vaginal delivery to shorten the second stage of labor. This study is a retrospective report. At the same time, oxytocin is not used in advance or widely in vaginal trial delivery women, resulting in a longer labor process even if oxytocin is used. This is also the direction of our further research.

## Figures and Tables

**Figure 1:** Comparison of labor process time between oxytocin group and nonoxytocin group: (a) first stage of labor, (b) second stage of labor, (c) total stage of labor.

**Figure 2:** Forest map of factors related to pregnancy success in VBAC pregnant women.

**Table 1:** Comparison of baseline clinical data between oxytocin group and nonoxytocin group.

Group	Number	Age (year)	Pregnancy times (times)	Production times (times)	BMI (kg/m^2^)	Gestational weeks of delivery (weeks)	Time from last delivery (months)	Thickness of lower uterine segment (mm)
Oxytocin group	42	32.91 ± 8.84	2.27 ± 0.44	1.16 ± 0.39	22.34 ± 3.87	39.60 ± 1.91	66.59 ± 12.46	2.53 ± 0.69
Nonoxytocin group	124	33.13 ± 8.29	2.19 ± 0.37	1.19 ± 0.33	21.64 ± 3.49	38.31 ± 1.70	64.89 ± 11.65	2.20 ± 0.55
*t*		0.17	−0.90	−1.39	0.13	−3.02	0.84	2.31
*P* value		0.91	0.44	0.28	0.35	0.00	0.48	0.04

**Table 2:** Comparison of labor time and pregnancy outcome between oxytocin group and non-oxytocin group.

Group	Number	First stage of labor (min)	Second stage of labor (min)	Total stage of labor (min)	Forceps assisted delivery (case)	Perineum incision (case)	Postpartum hemorrhage (case)	Fetal distress (case)	Neonatal asphyxia (case)	Entering NICU (case)
Oxytocin group	42	448.69 ± 110.44	40.90 ± 12.52	488.69 ± 110.48	31	24	7	8	0	2
Non oxytocin group	124	309.95 ± 97.10	32.91 ± 9.06	359.97 ± 87.08	97	62	19	33	1	17
*t*/*χ*^2^		−4.27	−5.89	−5.22	0.84	1.26	0.10	3.17	0.72	4.73
*P* value		0.00	0.00	0.00	0.33	0.26	0.87	0.06	0.89	0.04

The article "Influence of Oxytocin Usage and Dose Difference During Delivery on Pregnancy Outcome of VBAC Pregnant Women" was retracted in 2023. Reasons: unreliable results or conclusions; lack of ethics approval or compliance; concerns about the data; concerns about the peer review.

**Table 3:** Comparison of labor duration and pregnancy outcome in different oxytocin dose groups.

Group	Number	First stage of labor (min)	Second stage of labor (min)	Total stage of labor (min)	Forceps assisted delivery (case)	Perineum incision (case)	Postpartum hemorrhage (case)	Fetal distress (case)	Neonatal asphyxia (case)
Low-dose oxytocin group	22	418.72 ± 102.80	40.64 ± 15.52	458.58 ± 116.72	5	13	3	5	1
Medium dose oxytocin group	20	489.29 ± 127.33	39.90 ± 13.46	519.58 ± 130.82	7	11	4	3	1
*t*/*χ*^2^		−1.77	−0.26	−1.40	0.74	0.16	0.06	0.77	0.16
*P* value		0.26	0.80	0.34	0.38	0.25	0.82	0.36	0.94

**Table 4:** Univariate analysis of clinical data differences of VBAC pregnant women with different pregnancy outcomes.

Factors		Adverse outcome group (*n* = 87)	The normal group (*n* = 79)	*t*/*x*^2^	*P* value
Age (years)		33.34 ± 8.65	32.58 ± 7.87	0.590	0.556
Prenatal BMI (kg/m^2^)	≥30	22 (25.29)	45 (56.96)	17.257	<0.001
	<30	65 (74.71)	34 (43.04)		
Gestational age of delivery (weeks)	>40	31 (35.63)	11 (13.92)	10.324	0.001
	≤40	56 (64.37)	68 (86.08)		
Incision scar length (cm)		3.24 ± 0.88	3.31 ± 0.82	−0.529	0.598
History of vaginal delivery	Yes	16 (18.39)	41 (51.90)	20.608	<0.001
	No	71 (81.61)	38 (48.10)		
On admission, the uterine orifice is dilated (cm)	<6	46 (52.87)	20 (25.32)	13.127	<0.001
	≥6	41 (47.13)	59 (74.68)		
Admission	Labor in hospital	15 (17.24)	36 (45.57)	15.611	<0.001
	Nonclinical admission	72 (82.76)	43 (54.43)		
The birth weight of the newborn (kg)		3.35 ± 0.44	3.27 ± 0.39	1.235	0.219
The body weight of the previous newborn (kg)		3.24 ± 0.37	3.25 ± 0.34	0.361	0.718

**Table 5:** Factors related to pregnancy success in VBAC pregnant women.

Factors	B	S.E.	Wald	*P* value	OR	95% CI
Prenatal BMI <30 kg/cm^2^	0.882	0.372	6.258	0.006	0.515	0.051∼0.745
Gestational age ≤40 weeks	0.915	0.415	7.187	0.001	0.446	0.112∼0.618
History of vaginal delivery	0.783	0.316	5.866	0.003	0.294	0.142∼0.539
On admission, the uterine orifice is dilated	0.764	0.531	8.022	0.011	0.183	0.036∼0.278
Labor in hospital	0.629	0.559	7.269	0.002	0.372	0.159∼0.764

## Data Availability

The simulation experiment data used to support the findings of this study are available from the corresponding author upon request.
